The article "Effect of Bionic Nonsmooth Surface Vane on the Antiwear Characteristics of Double-Vane Pump" was published in 2022. Journal: Appl Bionics Biomech.

# Effect of Bionic Nonsmooth Surface Vane on the Antiwear Characteristics of Double-Vane Pump

**DOI:** 10.1155/2022/4442417

**Published:** 2022-04-20

**Authors:** Longbiao Ma, Yunqing Gu, Ke Xia, Jiegang Mou, Denghao Wu, Muhan Yan

**Affiliations:** ^1^College of Metrology & Measurement Engineering, China Jiliang University, Hangzhou 310018, China; ^2^Zhejiang Engineering Research Center of Fluid Equipment & Measurement and Control Technology, China Jiliang University, Hangzhou 310018, China; ^3^College of Mechanical Engineering, Zhejiang University of Technology, Hangzhou 310023, China

## Abstract

In order to improve the antiwear characteristics of the double-vane self-priming pump, the surface structure of the *Scapharca subcrenata* was extracted and reconstructed according to bionic principles. Three types of nonsmooth surface models were established at the outlet end of the suction surface of the vanes, which is the most severely worn in the double-vane pump. The external characteristics, pressure field distribution, wear area distribution, and wear degree of the volute and vanes at different concentrations of nonsmooth vane structure were investigated by numerical simulation to reveal the mechanism of the nonsmooth surface structure of the wear characteristics of the vanes. The results show that the head and efficiency of pumps with four different vanes decrease and the average wear rate increases as the particle concentration increases. The different vane structures have a very small effect on the wear resistance of the volute, but a larger effect on vane wear. The circular nonsmooth surface structure, which reduces the low pressure area of the inlet section of the impeller while ensuring a smaller drop in head and efficiency, produces the best antiwear effect and improves the antiwear performance of the double-vane pump.

## 1. Introduction

The double-vane self-priming pump is a type of centrifugal pump, which is an important equipment for transporting solid-liquid two-phase flow media and is used mainly in urban and industrial sewage containing suspended matter. As the core component of the pump, the impurities in the sewage continue to impact and break down the surface of the flowing parts during the discharge process, causing serious erosion of the flowing parts of the pump. The vanes can be impacted by the silt to form streaks, which destroy the surface shape of the vanes and affect the hydraulic performance of the pump [1, 2]. The resistance to wear therefore represents the performance of a double-vane pump [3].

Currently, improving the antiwear performance of flowing components relies on surface treatment techniques [4–6] and antiwear materials [7–9]. The surface treatment technology can directly improve the surface strength and hardness of the blade while providing a coating, but it is costly and has limitations. For antiwear materials, although the overall performance is very high, but only using the casting process leads to high process difficulties; it is difficult to ensure the accuracy of the blade and processing difficulties. Once the impeller is seriously worn, it can be impossible to repair, which will directly lead to a decline in the hydraulic efficiency of the pump.

Through evolution and natural selection over time, organisms have developed surface structures and functions that provide maximum adaptation and coordination for the environment in which they live. Engineering problems can therefore be helped by mimicking biological structures or by using artificial techniques to organismal biological functions. Bionic surface structures have attracted increasing attention to practical engineering due to their unique properties [10, 11], which also provide viable solutions to improving some of the properties of pumps with bionic nonsmooth structures. Currently, bionic nonsmooth surfaces have been used in pumps for applications such as anticavitation [12–14], vibration and noise reduction [15], and pressure pulsation reduction [16]. However, there are few studies on the wear resistance effects of these bionic nonsmooth surface structures for application in double-vane sewage pumps.

## 2. Bionic Prototyping and Structural Reconstruction

### 2.1. Biological Characteristics of *Scapharca subcrenata*

*Scapharca subcrenata* is a shellfish with a shell 40-50 mm long, consisting of calcium carbonate in the form of calcite. The anterior closed muscular scar is small and horseshoe shaped, while the posterior closed muscular scar is large and square. The shell is covered with a layer of dark brown fluff, and the surface and interior of the shell are white, with a thin layer of brown fluff. *Scapharca subcrenata* mainly inhabit soft mud bottoms or sandy bottoms in shallow waters (below 20 m).

During the long-term evolution of the *Scapharca subcrenata*, 30-35 prominent radial ribs were distributed over the surface of its shell to resist siltation. The structural features of the body surface are shown in Figure 1. Due to its grooved structure, the shell surface not only absorbs excess energy to relieve stress and improve biological resistance to scouring and abrasion but also generates vortex and cushion effects that reduce the abrasive strength and effective friction between the particles and the shell surface, further reducing the wear of the shell surface. Therefore, the application of this biological surface feature to improve the wear and scour resistance of the inner pump wall surface can effectively improve the boundary layer flow field of the wall surface, reduce the number of collisions, and improve the wear resistance.

The *Scapharca subcrenata* samples measured were from a seafood market in Hangzhou, China. The samples were selected based on the following criteria: adult grouper with a shell length of approximately 40 mm, a shell width of approximately 36 mm, and a shell height of approximately 36 mm, with the shell surface remaining intact. Meanwhile, to reduce measurement errors caused by impurities on the shell surface, all organic matter and other impurities were removed with a brush and clean water. Finally, 10 samples of grouper to be measured were obtained by forming dry bodies after air drying in a room at 25°C for 96 hours.

The microstructure of the shell surface was observed with an electron microscope, and the cross section of the grooves was found to resemble a trapezoidal structure. In measuring the surface structure of the shell, the middle groove of the shell was first found, and then, the sampling center was determined along the peak curvature point (PCP) of the shell at a distance of 20 mm from the PCP [17–19], as shown in Figure 1. Finally, electronic digital calipers are used to determine the width and height of the central groove and the spacing between adjacent grooves. To reduce errors, the data for each sample was measured five times. Using the groove width, height, and spacing as a set of data, 50 sets of data were obtained. The height, width, and spacing data for the measured samples were averaged separately to obtain a central groove depth of approximately 0.24 mm, a spacing of approximately 2.3 mm between the central groove and the adjacent groove, and a central groove width of approximately 0.42 mm.

### 2.2. Structural Reconstruction of Nonsmooth Surfaces

The bionic design has its origins in biology and is more advanced than biology. Based on the principles of bionics, the trapezoidal groove pattern on the surface of the fish is used as the biological prototype for the bionic structure. Combined with the current state of blade engineering, the bionic structure was reconstructed and extracted, and three bionic surface structures in line with the shape were constructed: triangular, circular, and rectangular. Based on the wear distribution of the centrifugal pump impeller, a triangular groove structure model, a circular groove structure model, and a rectangular groove structure model were reconstructed at the outlet end of the suction surface of the impeller. The effect of different shapes of nonsmooth structures on the antiwear performance of the double-vane pump was investigated. The bionic nonsmooth surface groove structure is shown in Figure 2, where *m* is the depth of the groove, *h* is the spacing between adjacent grooves, *θ* is the angle of the triangle, and *b* is the width of the rectangular groove. Considering the influence of the depth, width, angle, and alignment spacing of the nonsmooth surface structure on the blade strength, structure, and actual flow field, the parameters of the nonsmooth surface structure were improved, the alignment spacing of the nonsmooth surface structure was increased, and the model parameters *m* = 0.2 mm, *h* = 3 mm, *θ* = 90°, and *b* = 0.4 mm were determined.

## 3. Numerical Calculation Method

### 3.1. Modelling of Nonsmooth Surface Vane Structures

The 80ZW40-30 double-vane self-priming pump is used as a model pump during the study. The main performance parameters are pump flow rate *Q* = 40 m^3^/h, pump head *H* = 30 m, and pump speed *n* = 2800 r/min; structural parameters are impeller inlet internal diameter *D*_1_ = 80 mm, impeller inlet external diameter *D*_2_ = 164 mm, and number of vanes *Z* = 2.

In order to comprehensively analyze the erosion characteristics of the double-vane pump, a three-dimensional modelling of the fluid domain was carried out for the double-vane pump, as shown in Figure 3. Considering the combined effect of the gravity of the solid phase particles, virtual mass forces, interphase drag forces, and kinetic energy contained in the particles and turbulent eddies in the flow field, the main wear of the wheel blades is concentrated at the inlet end, the outlet end, and the middle of the suction surface, with the most serious wear at the outlet end [13, 20]. In addition, an excessive nonsmooth groove structure can seriously affect the distribution of the velocity and pressure fields inside the impeller, leading to a severe reduction in head and efficiency. Thus, the biomimetic nonsmooth surface structure was arranged around the suction end of the impeller near the outlet end region. The four different surface structures for the fluid domain model of the impeller are shown in Figure 4.

### 3.2. Mesh Division

The fluid domain was divided into unstructured meshes by the ICEM. Considering the complexity of the fluid flow field at the volute tongue, where severe flow field separation can occur, the mesh was encrypted at this location. The performance of a two-vane pump depends primarily on head and efficiency, and as the head is simpler and more intuitive to calculate than efficiency, the head is used as the basis for verifying mesh independence. When the calculation error is less than 0.8%, the scheme being tested is considered to be mesh independent, and the calculation error is calculated as shown in

(1) $$\begin{array}{c} \varepsilon =\frac{H_{n+1}-H_{n}}{H_{n+1}}\times 100\%, \end{array}$$

where *ε* is the calculation error and *n* indicates the scheme number.

The results of the grid independence analysis are shown in Table 1. The calculation error of scheme no. 4 is relatively small. Within the allowed error range, considering the calculation efficiency and workload, scheme no. 4 is finally chosen as the grid division of the calculation model.

### 3.3. Numerical Edge Strip Setting Parameter Model and Boundary Condition Setting

The standard *k-ε* turbulence model solves two independent transport equations to determine the turbulence length and time scales and has good robustness and reasonable prediction of large scale turbulence. Therefore, the standard *k-ε* turbulence model is chosen for the calculations. Taking into account the effects of interphase drag and slip velocity, the turbulent multiphase flow model uses the discrete particle model, which is currently the most used model for multiphase turbulence. The discrete particle model can be solved for the velocity, pressure, and erosion characteristics of particles at any point in the flow field. However, the application of the model requires that the volume fraction of solid particles should not exceed 12%, so the maximum volume fraction of solid particles under the study conditions is chosen to be 12% for the calculation. In terms of impeller wear, the Finnie erosion wear model predicts that the main areas of wear on the suction side of the blade are concentrated at the inlet and outlet ends, while the McLaury erosion wear model predicts that most wear occurs at the inlet, outlet, and middle of the suction side of the blade, which is much closer to the actual situation. The McLaury erosion wear model can be used to calculate the wear conditions at the walls of different flow components for different volume fractions of solid particles in the flow field and gives highly reliable predictions within the range of the discrete phase calculation. The model is formulated as follows [21]:

(2) $$\begin{array}{c} \text{WR}=2.17\times 10^{-7}\times F_{\text{p}}{v_{\text{p}}}^{2.41}F\left(\alpha \right), \end{array}$$

(3) $$\begin{array}{c} \text{ER}=\sum \frac{m_{\text{p}}\text{WR}}{{tA}_{\text{cell}}}, \end{array}$$

where WR is the wear weight loss rate and *F*_p_ is the particle shape coefficient. *F*(*α*) is the impact angle function, which is often expressed as a piecewise polynomial [22]. For spherical particles, *F*_p_ = 1; *V*_p_ is the solid phase velocity, m/s; *α* is the particle incidence angle, deg; ER is the wear rate, kg/s^2^·m; *M*_p_ is the mass of single solid particle, kg; *T* is the total collision time, s; and *A*_cell_ is the wall mesh area of the computing unit, m^2^.

According to equations (2) and (3), it can be concluded that the wall erosion wear rate is related to three parameters including particle collision times, incident velocity, and angle of solid particles.

The solid-liquid two-phase flow medium is water containing sand, and the solid particles are mainly composed of SiO_2_. SiO_2_ density *ρ*_p_ = 2650 kg/m^3^, and SiO_2_ particle size *r* = 0.5 mm. Solid-liquid two-phase flow media with particle mass concentrations (density) of 0, 10, 30, 50, 70, and 90 kg/m^3^ were used under different study conditions. The corresponding volume fractions of gravel particles in the transport media under different conditions are 0%, 0.377%, 1.132%, 1.887%, 2.642%, and 3.396% according to equation (4). Using the SIMPLEC pressure-velocity coupling algorithm, the inlet boundary condition was set to velocity inlet and the outlet boundary condition to free outflow. A slip grid was chosen for some of the impeller fluid domains, and a static coordinate system was chosen for the other fluid domains. The walls are slip-free; the reference pressure is standard atmospheric pressure; the convergence accuracy is 10^−4^. The inlet is the discrete, phase is the inlet, and the outlet is the only outlet of the discrete phase, while the other walls are set as reflective walls.

(4) $$\begin{array}{c} \varphi =\frac{\rho }{\rho_{\text{p}}}\times 100\%. \end{array}$$

In addition, for the numerical calculation of the solid-liquid two-phase turbulence, we made the following assumptions: (i) the liquid medium water is the first phase, the solid particles sand is the second phase, both are uniform in size and spherical, and both phases have no phase change; (ii) the solid particles are uniformly distributed in the liquid fluid, and the medium density is uniform.

## 4. Analysis of Pump Performance of Nonsmooth Surface Vane Structure

### 4.1. Analysis of External Characteristics

Double-vane pump in the transport of solid-liquid two-phase flow media, its efficiency and head way and a single clear water media, head formula is shown in

(5) $$\begin{array}{c} H_{\text{m}}=\left(1-\varphi \right)\frac{P_{\text{out}}-P_{\text{in}}}{\rho g}, \end{array}$$

where *H*_m_ is the pump head when conveying solid-liquid two-phase flow medium, m; *φ* is the solid phase volume fraction; *P*_in_ is the pump inlet pressure, Pa; *P*_out_ is the pump outlet pressure, Pa; and *ρ* is the density of solid-liquid two-phase flow, kg/m^3^.

The efficiency formula of double-vane pump for conveying solid-liquid two-phase flow medium is shown in

(6) $$\begin{array}{c} \eta =\frac{\rho q_{\text{v}}{gH}_{\text{m}}}{3600\times 1000N}, \end{array}$$

where *η* is hydraulic efficiency; *Q*_v_ is the volume flow rate, m^3^/h; and *N* is the shaft power, kW.

Figure 5 shows the head curves of the double-vane pump at different concentrations. As can be seen in Figure 5, the head of all four vanes of the double-vane pump decreases as the mass concentration of the particles increases. When sand particles are added to the fluid, the sand particles collide with the surface of the flowing parts and with each other during transport, thus consuming the total energy in the flow field and causing the head to decrease. As is known from Figure 5, pumps with smooth vanes have the highest head. When the medium is water, the head value is 31.7 m, which is higher compared to the rated head of 30 m. This is because only the volute chamber and impeller are considered in the numerical simulation and energy losses not related to the wear of the flow components in the gas-liquid separation chamber and the return orifice are ignored. The simulated values of the head are therefore within the permissible margin of error.

The pump head of the circular nonsmooth vane is 2% lower than that of the smooth vane, and its head is similar to that of the smooth surface vane. The head of triangular nonsmooth vane and rectangular nonsmooth vane decreases greatly, and the head of rectangular nonsmooth vane decreases the most compared with smooth vane.

Figure 6 shows the efficiency curve of the double-vane pump at different concentrations. It can be seen from Figure 6, with the increase of particle mass concentration, the variation trend of the efficiency of the double-vane pump of four different vanes decreased. The efficiency of the double-vane pump with smooth vane is the highest; the efficiency of the circular nonsmooth vane is close to that of the smooth vane and decreases by less than 1%. The efficiency of the double-vane pump with rectangular nonsmooth vane is the lowest, and the decrease of efficiency of the double-vane pump with smooth vane is less than 3%. This is due to the recesses of the rectangular and triangular structures, which do not conform to the flow characteristics of the fluid and are prone to vortexes. Under the action of the vortex, the two-phase flow rotates and collides in the groove, consuming its own energy. Meanwhile, rectangular structure has two walls perpendicular to the direction of motion of the medium. In the process of fluid flow, the flow area locally undergoes two stages of sudden expansion and sudden reduction, leading to redistribution of fluid velocity. This process not only intensifies the internal friction of the fluid but also causes the backward and forward collision of the fluid particles, which increased the turbulence in the fluid and led to excessive energy loss and head and efficiency reduced. Therefore, it can be learned that the head and efficiency of the rectangular nonsmooth vane are the lowest. However, the circular surface of a circular nonsmooth vane can better conform to the law of fluid flow without right angles or excessive bends, so its head curve and efficiency curve are similar to those of a smooth vane.

### 4.2. Pressure Field Distribution Analysis

Figure 7 shows the pressure cloud of the cross section of the double-vane pump with four different vanes for *ρ* = 0 kg/m^3^. By analyzing the internal pressure field of the double-vane pump without adding solid particles, the effects of different shapes on the flow field inside the pump body were studied. The influence of the change of pressure field on the antiwear performance was further expounded. Figure 7 shows that under the design conditions of clean water, namely, the particle concentration *ρ* = 0 kg/m^3^, the overall flow state inside the impeller passage is stable and the pressure distribution is uniform. Because the vane rotation will work on the incoming fluid and the kinetic energy is converted into pressure energy, the pressure distribution law of the flow field inside the impeller increases from the inlet end to the outlet end. Through observation, the blade was found to be at the water end of the pressure of the lowest easily occurring cavitation. At the same time, because there is a low pressure area at the inlet end of the vane, sand-containing water will cause impact on the vane. The pressure distribution in the internal section of impellers with different vanes is different, and the low-pressure area in Figures 7(b) and 7(d) is more obvious, because the structure of rectangular and triangular nonsmooth surfaces does not conform to the flow state of the internal fluid. Compared with Figures 7(b) and 7(d), the low-pressure area in Figures 7(a) and 7(c) is relatively reduced, because the smooth surface and circular nonsmooth surface are consistent with the flow state of the fluid on the vane surface. The four kinds of vane pressure double-vane pump volute flow field distribution are relatively uniform, which means less nonsmooth surface structure can affect the volute pressure distribution, and the stress distribution inside the volute is mainly related to the diffusion section. Along with the increase of the diffusion section of the cross-sectional area of the speed of the fluid can be converted into pressure, to maximize the pressure at the exit of the spiral case. There is a local high pressure area at the volute tongue, which is due to the existence of a small gap at the septum and the rotating blade at the end of the water causing a relatively strong static and dynamic interference, changing the flow of liquid state.

Figure 8 shows the pressure distribution for clouds for four different vane surface configurations for *ρ* = 0 kg/m^3^. Figure 8 shows that the pressure increases continuously from the inlet end of the impeller to the outlet end, with the lowest pressure at the inlet end and the pressure at the pressure surface being greater than the pressure at the suction surface, which is in accordance with the basic operating principle of centrifugal pumps. Only when the pressure on the suction surface of the vane is less than that on the pressure surface can the fluid medium continue to flow into the pump.

By comparing the four different surface structures of the vane, it was found that the pressure distribution on the suction surface of the smooth vane and the circular nonsmooth vane is similar and increases uniformly, while the low-pressure area on the suction surface of the rectangular nonsmooth vane and the triangular nonsmooth vane near the inlet end is relatively large.

### 4.3. Analysis of Wear Resistance

#### 4.3.1. Antiwear Performance of Volute

Figure 9 shows the average wear rate-particle concentration histogram for smooth blades and three nonsmooth blade worm gears of different configurations. As the concentration of sand particles increases, the average wear rate of the four blades increases. The results show that when the concentration of particles in the medium is excessively high, the worm shell surface is severely eroded, causing the worm shell to be the first to fail and reducing the service life of the two-vane pump. When the concentration of particles is equal, the average wear rate of the smooth vane worm shell is compared with the average wear rate of the nonsmooth vane worm shells of three different configurations. It was found that the average wear rate of the smooth vane worm shell was slightly greater than that of the three nonsmooth vane worm shells, but there was no significant difference. When the particle concentration *ρ* = 90 kg/m^3^, the average wear rate difference is the largest, and the maximum difference between the average wear rate of the worm shells with smooth blades and rectangular nonsmooth blades is 0.39%, which is basically negligible. This shows that although the average wear rate of the worm shell increases with increasing particle concentration, it is largely unaffected by the bionic nonsmooth surface structure of the blade surface.

#### 4.3.2. Antiwear Performance of Vane

Figure 10 shows the curves of the average wear rate and particle concentration for smooth and nonsmooth blades of three different configurations. The average wear rate of the four blade surfaces increases linearly with increasing particle concentration [23]. The overall average wear rate compared to particle concentration was rectangular nonsmooth vane > triangular nonsmooth vane > smooth vane > circular nonsmooth vane. The circular nonsmooth vane had the lowest average wear rate, with a relatively flat trend compared to the other three blades. At a particle concentration of *ρ* = 90 kg/m^3^, the average wear rate for blades with circular nonsmooth surfaces is approximately 56% lower than the average wear rate for smooth surfaces.

Figure 11(a) shows a cloud plot of the wear rate distribution on the smooth vane wall for different particle concentrations. When the vanes of the two-vane pump are smooth, the wear range gradually expands as the particle concentration increases. When the particle concentration is less than 50 kg/m^3^, the pitting corrosion on the vane wall is randomly distributed onto the suction surface and not connected to each other. The wear area is mainly concentrated on the suction surface near the inlet end of the blade and the suction surface near the outlet end of the blade, and the area connected to the back cover is less worn. When particle concentration is greater 50 kg/m^3^, the wear rate on the blade walls increases significantly and interconnects, forming a worn zone distributed over the entire end portion of the blade suction surface.

Figure 11(b) shows a cloud plot of the distribution of wall wear rates for triangular nonsmooth vanes with different particle concentrations. When the particle concentration *ρ* = 10 kg/m^3^, there are scattered erosion zones at the inlet end of the blade and in the nonsmooth area. As the particle concentration increases, the wear between the inlet end of the blade and the nonsmooth area deepens and the “wear zone” evolves into a “wear zone band.” As the particle concentration increased from 70 kg/m^3^ to 90 kg/m^3^, the wear area of the blade inlet face did not change significantly, indicating that the wear surface did not extend into the lateral area as the particle concentration increased. However, the increase in wear rate indicates that in practice, the area is being worn more severely.

Figure 11(c) shows a cloud plot of the wall wear rate distribution of a circular nonsmooth blade for different particle concentrations. When the particle concentration *ρ* = 90 kg/m^3^, the wear area is distributed in three parts: the inlet end of the blade, the nonsmooth zone of the blade, and between the suction end of the blade. As the particle concentration increases, the wear in the nonsmooth zone does not change significantly, but the wear in the tip area of the suction surface between the inlet end and the nonsmooth zone deepens significantly, and the shape of the wear zone gradually extends from a lumpy shape at the beginning to a strip shape.

Figure 11(d) shows a cloud plot of the wall wear rate distribution for rectangular nonsmooth blades with different particle concentrations. As the particle concentration increases, the shape of the wear area changes from blocky to stripy. This indicates that when the particle concentration is overly large, the suction surface of the blade wall will erode the strip-shaped wear area due to the impact and collision of solid particles on the wall, which will seriously affect the stress distribution of the blade and lead to deformation, fracture, or even failure of the blade.

Under the same particle concentration conditions, the degree of wear of the smooth vane walls significantly differs from that of the three nonsmooth vanes. Combined with the comprehensive analysis of the average wear rate-particle concentration curve in Figure 10, the degree of wear of the circular nonsmooth vanes is small when the particle concentration *ρ* = 90 kg/m^3^. The wear area is divided into three parts: the inlet end of the blade, the nonsmooth area of the blade, and the end area between the suction surfaces of the blade. Although the rectangular and triangular nonsmooth structure plays a role in dispersing the stress to a certain extent, the wear area is concentrated and the degree of wear is severe.

### 4.4. Antiwear Mechanism

According to the above analysis, the circular nonsmooth surface blade structure has the best antiwear characteristics compared to the other two bionic nonsmooth structures. The reason for this is that the existence of circular nonsmooth structures causes a low velocity vortex zone to form inside the groove. The fluid at the bottom of the groove is in the same velocity direction as the field, while the velocity direction inside the groove is opposite to the velocity direction of the groove and is less than the fluid velocity at the bottom of the groove. This internal reverse vortex plays the role of the “air cushion” [24]. The solid line is the flow line of the liquid phase, and the dashed line is the trajectory of the solid phase. Smooth zones in the solid phase particles directly with the blade wall contact and collision, the formation of wear zones, while the circular nonsmooth zone due to the role of vortex, can neutralize the impact of solid phase particles, change the size and speed direction of the particles, and reduce the frequency of particle and blade wall distribution of the impeller. Compared to the other two nonsmooth structures, the circular nonsmooth vanes reduce the low-pressure area in the inlet section of the double-vane pump and direct collisions and to a certain extent improve the blade wall antiwear performance.

## 5. Conclusion

1. Based on bionic principles, the groove surface structure of the *Scapharca subcrenata* has been refined. Three bionic nonsmooth surface models, circular, rectangular, and triangular, are introduced to the outflow end of the suction surface of the most severely worn vane by means of a double-vane pump
2. As the particle concentration increases, the head and efficiency of the four different vane types of twin vane pumps decrease. The smooth twin vane has the highest efficiency under the same particle concentration conditions. The efficiency of the circular nonsmooth vane is closer to that of the smooth vane and decreases in the permissible range
3. The nonsmooth surface construction has a scarcely noticeable effect on the pressure distribution of the volute, but not on the pressure
4. The average wear rate of the four types of two-vane pumps increases with increasing particle concentration. At the same particle concentration, the average wear rate of the circular nonsmooth vane is lower than that of the other configurations. For different parts of the pump, the nonsmooth structure improves the antiwear conditions in different ways. For the volute structure of the pump, the maximum difference in wear rate is less than 0.39%, which is a small improvement. However, there is a significant impact on the wear performance of the vanes. The presence of circular grooves in the nonsmooth structures allows the vane surface to form a reflux zone at low speeds, which reduces the average wear rate of the vanes by around 56% by reducing the frequency probability of direct collision of the particles and the vane wall and improves the antiwear performance significantly

## Figures and Tables

**Figure 1:** Surface structure of *Scapharca subcrenata*.

**Figure 2:** Schematic diagram of a bionic nonsmooth surface structure.

**Figure 3:** Schematic diagram of fluid domain.

**Figure 4:** Impeller fluid domain with four different surface structures.

**Figure 5:** Particle concentration-head curve of a double-vane pump.

**Figure 6:** Particle concentration-efficiency curve of a double-vane pump.

**Figure 7:** Cross-sectional pressure clouds of four vane double-vane pumps at *ρ* = 0 kg/m^3^.

**Figure 8:** Cloud plot of pressure distribution of vanes at *ρ* = 0 kg/m^3^.

**Figure 9:** Average wear rate of worm shell at different vanes—particle concentration histogram.

**Figure 10:** Average wear rate particle concentration curve of double-vane pump vanes with different structured vanes.

**Figure 11:** Nephogram of four kinds of blade wall wear rate distribution with different particle concentrations.

**Table 1:** Mesh independence analysis results.

Item no.	Inlet pipe	Outlet pipe	Impeller	Snail shell	Simulated values of head (m)	Calculation errors
1	213475	85446	621454	623145	32.71	
2	293346	103571	841546	721354	32.23	1.46%
3	357984	137518	945644	846543	31.91	0.99%
4	463407	152529	1278468	1174594	31.70	0.65%
5	557259	207628	1572137	1446483	31.76	0.19%

## Data Availability

The data used to support the findings of this study are available from the corresponding author upon request.
